# Design of Water Quality Monitoring System in Shaanxi Section of Weihe River Basin Based on the Internet of Things

This article has been retracted.

**DOI:** 10.1155/2022/3543937

**Published:** 2022-07-21

**Authors:** Tianjiao Dang, Jifa Liu

**Affiliations:** School of Marxism, Chang'An University, Xi'an 71000, China

## Abstract

Monitoring environmental water quality in an efficient, cheap, and sustainable way can better serve the country's strategic requirements for water resources and water ecological protection. This paper takes the Shaanxi section of the Weihe River Basin as a pilot project and aims to use the Internet of Things technology to develop water quality monitoring sensors, so as to realize the construction of low-cost, high-reliability water quality monitoring demonstration applications. First of all, we established the design of the water quality collection terminal, designed the low-power water quality sensor node, supported the Internet of Things protocol and the collection of various water quality parameters, and used networking for data transmission. Secondly, we use the ant colony algorithm-based system clustering model to obtain a cluster map of water quality monitoring tasks in a certain section of the Weihe River Basin. We take the task clustering graph as an example for analysis, optimize the monitoring model through the ant colony algorithm, and obtain the weight of the optimization index. The weight of the scheduled task limit of the monitoring point becomes larger, so the release of the monitoring task mainly affects the limit of the scheduled task of the monitoring point. Through the above work, we designed and implemented a set of online water quality monitoring system based on the Internet of Things and data mining technology. The system can provide reference for large-scale water resource protection and water environment governance.

## 1. Introduction

Whether the water quality monitoring industry can develop stably and continuously is an important foundation for national economic and social development. China's water resources are seriously uneven in terms of regional distribution and seasonal distribution [1, 2]. The availability of highly limited water resources is the responsibility of our entire society [3]. By monitoring and analyzing comprehensive indicators that can reflect water quality conditions, such as temperature, pH value, suspended solids, turbidity, flow rate, and flow rate, as well as monitoring and forecasting floods and droughts, the water conservancy department is responsible for forecasting water conditions and making decisions [4–6]. The most important feature of the automatic water quality monitoring system is that it can monitor the water quality in a timely, accurate, and effective manner. However, the traditional hydrological monitoring technology is backward, the sampling capacity is insufficient, and the information is collected and processed almost manually. Constrained by various conditions, the emergency treatment capacity is not high, and the on-site monitoring and management is weak [7–9]. The rapid development of microelectronic technology, communication technology, computer technology, etc. makes us put forward higher requirements for hydrological work. Improving the level of information transmission, realizing remote monitoring of water quality, timely grasping the water quality status of major river basins, and improving emergency monitoring capabilities are all important for water quality monitoring [10, 11].

With the growth of population and the development of industrial and agricultural production, residents' demand for water is increasing, so the shortage of water resources and serious water pollution are considered a severe test for water quality monitoring. The automatic water quality monitoring system is based on monitoring the comprehensive indicators of water pollution and some specific items. By setting up thousands of monitoring stations with continuous automatic monitoring instruments in a water system, the water pollution status of the area can be monitored continuously and automatically [12]. At present, this type of water quality automatic monitoring system is mainly used to detect the water quality of a certain water area. In Europe, the United States, and other countries, a large number of water quality analyzers with various parameters began to appear in the 1980s. Japan, the United States, the Netherlands, and the United Kingdom have already used them on a considerable scale and have become very common [13–15]. Thousands of wireless interconnected monitoring stations are set up in a certain area, and the stations are based on comprehensive indicators of water pollution such as turbidity, electrical conductivity, chemical oxygen demand, pH value, and water temperature. These monitoring stations are distributed by the central control system. Under the unified and coordinated work, the water pollution status in the designated area can be measured accurately in real time [16]. Finally, the collected water quality information can be transmitted through carriers such as GPS global satellite positioning system. Although Japan has a small land area, it has developed earlier in the research and development of water quality monitoring systems. Their main advantages lie in the high degree of automation and the relatively high degree of integration of modules [17].

IoT has vast applications, and it can be used in monitoring water quality to provide clean water and control the wastage of natural resources. The best aspect of IoT is that it is easy to maintain and use, and because it is connected to the internet, it provides real-time control. The real-time control process can be achieved by using wireless sensors and sending data through sensors to the cloud. This process will be efficient, and in this way, the manual cost of monitoring can be eliminated using a digital-based IoT system. This will improve the management quality and efficiency [18].

This paper mainly describes the overall scheme of designing an online water quality monitoring system, formulates some software and hardware design principles, and briefly introduces key technologies such as Internet of Things networking and data analysis. The corresponding river data are collected by the sensors laid in the river, and the data collected by the sensors are integrated on the built network and transmitted to the cloud, and the cloud uploads the collected data to the background management system. The relevant personnel can view the corresponding data through the background management system, so as to have a clearer understanding of the river situation [19].

## 2. Related Overview

The Weihe River is the largest river in Guanzhong and a first-class tributary of the Yellow River. The Weihe River Basin has a total area of 135,000 square kilometers. It flows through Shaanxi, Gansu, and Ningxia provinces and plays a vital role in the development of industry and agriculture on both sides of the river [18]. Among them, the basin area in Shaanxi is 67,100 square kilometers, accounting for 50% of the total area of the Weihe River Basin. Now the Weihe River is the largest river flowing through Guanzhong in Shaanxi Province and is the “mother river” of the Guanzhong area. With the rapid economic development in Central Shaanxi, the production and domestic sewage (waste) water discharge along the Weihe River has increased year by year.

With the rapid economic development in Central Shaanxi, the discharge of domestic sewage and industrial wastewater along the Weihe River is also increasing year by year. Due to the intensification of governance, most polluting enterprises have built water pollution control facilities, but there are still some enterprises that are still unable to discharge stably up to the standard for a long time [20, 21]. Therefore, for natural rivers, even if all industrial wastewater is treated and discharged up to standard, the concentration of pollutants in wastewater is still high. With the acceleration of urbanization and the continuous increase of population, the increase of domestic sewage discharge is still the main source of pollution to the water quality of the Weihe River Basin. In 2007, the urban sewage treatment rate along the Weihe River was less than 40%, but more than 60% of the untreated domestic sewage was directly or indirectly discharged into the Weihe River [22]. The existing water quality monitoring methods all have some shortcomings, which cannot meet the needs of real-time online monitoring of water quality parameters in large areas of water, complex terrain waters, and waters that are difficult for humans to reach. At the same time, the cost-effectiveness of the existing scheme is low, and the effective monitoring and management of the complex water environment cannot be realized. In addition, the above monitoring methods only involve water quality monitoring and do not pay attention to the summary and analysis of test data. Therefore, the comprehensive analysis level of water environmental quality is relatively low, and it cannot be well applied to environmental management services.

## 3. Water Quality Detection in the Shaanxi Section of the Weihe River

The existing lake water environment monitoring system is only responsible for collecting the water quality parameters of the water area to be measured and cannot realize automatic and intelligent management from data collection to water quality analysis [23, 24]. In addition, although scholars have tried many methods to realize the analysis and diagnosis of water quality, they have not reasonably expressed the relevant knowledge in the field of water environment, so the evaluation results obtained are difficult to be understood by users [25]. At the same time, the traditional monitoring methods of water quality testing and water quality evaluation are isolated from each other, which increases the difficulty of water environment management. The water quality monitoring system based on the Internet of Things architecture proposed in this paper can not only collect water quality data but also integrate an intelligent decision-making module, which can monitor, evaluate, and predict the water quality of the lake to be measured in real time, thereby improving the management level of the lake water environment [26].

### 3.1. Design of IoT Monitoring System

In this paper, the system is divided into perception convergence layer and application layer, which consists of three parts: water quality monitoring terminal, water quality gateway, and water quality monitoring center. Facing the complex environment and wide range of monitoring waters, the system adopts the idea of divide and conquer, dividing the whole water area into multiple monitoring subnetworks [27, 28]. When the system is running, the monitoring terminal establishes its own water quality monitoring network in the target water area, and the water quality gateway uploads the water quality data through the backbone transmission network, completes the data aggregation and management in the monitoring center, and finally realizes the online water quality monitoring of the target water area.  Figure 1 shows the overall design framework of the water quality monitoring system.

The water quality monitoring terminal is an execution device on the system perception and convergence layer, which is widely deployed in the target waters, and its core task is the online collection and transmission of water quality information [29]. Several monitoring terminals use ZigBee technology to dynamically set up water quality monitoring subnetworks. During operation, the terminals collect pH, water temperature, conductivity, and dissolved oxygen parameters of the water body according to system instructions and realize a large amount of water quality data in-network aggregation.  Figure 2 depicts a schematic diagram of the water quality monitoring nodes.

As the communication relay of monitoring subnet and monitoring center, water quality gateway has two important functions. First, it is responsible for monitoring the protocol conversion between the proprietary wireless network of the subnet and the external IP network, completing remote data transmission and command parsing and forwarding. Second, it assists the monitoring terminal to complete the tasks assigned by the system and monitor its equipment status, so as to realize the autonomous management of the monitoring subnetwork. The water quality monitoring center is the management center of the system, which is deployed on the remote PC for management personnel to use. Based on remote data access and database operation, the monitoring center has basic functions such as water quality data statistics, equipment monitoring and control, historical data query, and automatic alarms. A water quality monitoring point optimization model with ant colony algorithm as the core is embedded in the monitoring center to better combine data storage and data analysis, thereby improving system integration.

### 3.2. Monitoring Task Optimization

#### 3.2.1. Systematic Clustering of Monitoring Points

Systematic clustering is to first classify *n* samples into one class and calculate the distance between them. Select two samples with the smallest distance and classify them into a new class, calculate the distance between the new class and other samples, and then select the two samples with the smallest distance to be combined into one class, so that one class is reduced each time until all samples become one class. This paper adopts the shortest distance method to define the distance between classes. Let *d*_*ij*_ represent the distance between the *i*th sample and the *j*th sample, and define the distance between the two classes to be represented by the distance between all samples between the two classes.

(1) $$\begin{array}{c} D_{uv}=\min\left\{d_{ij}\right\},\\ x_{i}\in G_{u},\\ x_{j}\in G_{v}, \end{array}$$

where *X*_*i*_ ∈ *G*_*u*_ indicates that the *i*th sample belongs to class *G*_*u*_, *X*_*j*_ ∈ *G*_*u*_ indicates that the *j*th sample belongs to class *G*_*v*_, and *D*_*uv*_ is the smallest distance between all samples in the two classes.

The following basic steps are generally required when applying a systematic clustering method. First, the distance (Euclidean distance) is specified, and the distance between each sample is calculated first and recorded in the classification distance symmetry table. Set to *D*_*uv*_ by choosing the shortest distance obtained in the first step. Compute the distance between the new class *D*_*r*_ and the other classes.

(2) $$\begin{array}{c} D_{rk}=\underset{\begin{array}{c} i\in G_{r}\\ j\in G_{k} \end{array}}{\min}\left\{d_{ij}\right\}\\ =\min\left\{\underset{\begin{array}{c} i\in G_{r}\\ j\in G_{k} \end{array}}{\min}d_{ij},\underset{\begin{array}{c} i\in G_{v}\\ j\in G_{k} \end{array}}{\min}d_{ij}\right\}. \end{array}$$

We delete the *u*th row and *v*th column in *D* (0) and add the *r*th row and *r*th column to obtain a new distance symmetry table, denoted as table, which represents the distance table after one clustering. Under the *D* (1) table, indicate which two categories are included in D(r). The table can be obtained by repeating the clustering work similar to *D* (0) for *D* (1) in the steps from the second to the fourth step. This is a new classification distance symmetry table obtained by secondary clustering.

### 3.3. Ant Colony Algorithm Optimization

Let the total number of ants in the ant colony be *m*, *d*_*ij*_(*i*, *j*=1,2,…, *n*) represent the distance between tasks *i* and *j*, and *b*_*i*_(*t*) represent the number *m*=∑_*i*=1_^*n*^*b*_*i*_(*t*) of ants in task *i* at time *t*. *τ*_*ij*_(*t*) represents the amount of information between tasks *i* and *j* at time *t*. At the initial moment, the amount of information on each path is equal. Ant *k*(*k*=1,2 …, *m*) decides the transfer direction according to the amount of information on each path during the movement. *p*_*ij*_^*k*^(*t*) represents the probability that ant *k* is transferred from task *i* to task *j* at time *t*.

(3) $$\begin{array}{c} p_{ij}^{k}\left(t\right)=\left\{\begin{array}{cc} \frac{\tau_{ij}^{\alpha }\left(t\right)\eta_{ij}^{\beta }\left(t\right)}{\sum_{r\in {\text{allowed}}_{k}}\tau_{ir}^{\alpha }\left(t\right)\eta_{ir}^{\beta }\left(t\right)}, & j\in {\text{allowed}}_{k},\\ 0, & \text{otherwise,} \end{array}\right. \end{array}$$

where allow*d*_*k*_={0,1,…, *n* − 1} − *tabu*_*k*_ represents the set of task points that ant *k* is allowed to walk through in the next step. After *n* moments, the ants can complete all tasks and complete a cycle. The path taken by each ant is a solution.

(4) $$\begin{array}{c} \tau_{ij}\left(t+1\right)=\left(1-\rho \right)\cdot \tau_{ij}\left(t\right)+\Delta \tau_{ij}, \end{array}$$

where *ρ* ∈ (0,1) is the evaporation factor.

(5) $$\begin{array}{c} D\left(x_{i},\mu_{k}\right)=\sqrt{\sum_{j=1}^{d}{\left(x_{ij}-\mu_{kj}\right)}^{2}},\;\left(x_{i}\in c_{k}\right). \end{array}$$

The initial starting point of each monitoring point is placed in the current solution set, and each monitoring point *k*(*k*=1,2,…, *m*) is moved to the next vertex *j* according to the probability *Z*_*k*_(*k*=1,…, *m*), and the vertex *j* is placed in the current solution set. Calculate the objective function value of each monitoring point and record the current best solution after running the program each time. If the number of iterations is predetermined and there is no degenerate behavior, the current optimal solution is output.  Figure 3 depicts the ant colony algorithm optimization flowchart.

It can be concluded from the new detection model that when the detection tasks are packaged and released in a centralized manner, the weight of the limited quota of monitoring points becomes larger, that is, this factor is the main indicator factor in the new pricing model.

## 4. Water Quality Monitoring Model Test

This paper aims to develop a set of online monitoring system for real-time monitoring and analysis of lake water quality. We have described in detail the software and hardware design scheme for the realization of system functions and the specific realization of the water quality evaluation and prediction module based on ontology and grey theory. In order to ensure the normal operation of the lake water quality monitoring system, it is necessary to ensure the normal operation of each submodule that constitutes the system. Therefore, various functions specified by the system and various performance parameters of the system should be verified to determine the lake water quality monitoring designed in this paper. The latitude and longitude data of the relevant monitoring points in the Weihe River Basin are brought into the above formula, and then according to the five basic steps of systematic clustering, the data table and task clustering diagram generated in the clustering process can be obtained.  Table 1 shows the clustering results of monitoring point locations.

For monitoring nodes, the data collection accuracy is also affected by factors such as climate and environment in practical applications, as well as the accuracy of the sensor itself. Therefore, the accuracy of data received by the remote monitoring center will also be affected accordingly. Since the water quality sensors used in the system are also different in accuracy, this paper intends to compare the collected data with the standard data and calculate the indication error and repeatability error. Due to limited conditions, the data collection accuracy is only evaluated in the laboratory environment. This paper only verifies the acquisition accuracy of the existing pH sensor, temperature sensor, conductivity sensor, and dissolved oxygen sensor. The indication error and repeatability error of the sensor under different water quality conditions are calculated, as shown in Table 2.

It can be seen from Table 2 that the indication error of the pH value collected by the water quality testing system is not higher than 0.1PH, and the repeatability error is not higher than 0.05PH. The temperature indication error is not higher than 1.0°C, and the repeatability error is not higher than 0.3°C when it is lower than 40°C. The indication error of conductivity is not higher than 3.0%FS, and the repeatability error is not more than 1.0%FS. The indication error of dissolved oxygen does not exceed 5.0%FS, and the repeatability error does not exceed 2.5%FS. The above test data show that although the water quality monitoring system developed in this paper has certain errors in data collection, it basically meets the accuracy requirements of the river water quality monitoring system.

## 5. Conclusion

The intelligent management platform scientifically analyzes the current environmental data, generates various scenarios operated by the platform operators, and adjusts and controls the water quality and environment in real time to ensure that water pollution is effectively dealt with in a timely manner. Online monitoring of water quality can better promote the real-time, intelligent, and unmanned monitoring of water quality. With the help of the Internet of Things technology, the data of each sensing terminal are transmitted to the platform in real time. The platform systematically completed the development of water management institutions and rivers and lakes, and established an online water quality monitoring system. Through this platform, we can conduct time-sharing research and processing on relevant data, and give corresponding processing results. Experiments have proved that it is feasible and effective to realize water quality monitoring through the Internet of Things. By building a data acquisition network, the acquisition central station is used to collect and upload data, and the network transmits, collects, and stores the data by the host computer software. The whole system has low labor maintenance cost, high collection efficiency, and large data capacity, which is conducive to analysis and statistics. The whole system has been tested and debugged to achieve the expected effect, providing real-time and effective data for water quality monitoring, and the cost is low.

## Figures and Tables

**Figure 1:** Overall design framework of water quality monitoring system.

**Figure 2:** Schematic diagram of water quality monitoring nodes.

**Figure 3:** The flowchart of ant colony algorithm optimization.

**Table 1:** Clustering results of monitoring point locations.

Cluster table						
Order	Cluster composition		Coefficient	First occurrence of phasic cluster		Next level
	Cluster 1	Cluster 2		Cluster 1	Cluster 2	
1	36	37	0.000	0	0	12
2	16	17	0.000	0	0	20
3	26	30	0.000	0	0	5
4	28	29	0.000	0	0	6
5	26	27	0.000	3	0	6
6	26	28	0.000	5	4	10
7	12	21	0.000	0	0	10
8	10	11	0.000	0	0	11
9	2	3	0.000	0	0	33
10	12	26	0.001	7	6	16
11	10	14	0.001	8	0	19
12	20	36	0.001	0	1	13
13	20	31	0.001	12	0	26
14	4	15	0.001	0	0	17
15	23	35	0.001	0	0	26
16	12	24	0.001	10	0	22
17	4	25	0.002	14	0	27
18	9	19	0.002	0	0	24
19	10	13	0.003	11	0	28
20	8	16	0.003	0	2	27

**Table 2:** Indication error and repeatability error under different water quality conditions.

Test items		Theoretical value	Detection value				Error	Repeatability
Test 1	pH	6.0	5.94	6.14	6.09	6.05	−0.003	0.11
		6.5	6.39	6.45	6.37	6.67	−0.019	0.12
		7.0	6.83	6.88	7.15	6.82	−0.03	0.16

Test 2	Temperature (°C)	15	14.6	14.38	15.43	15.09	0.018	0.44
		20	19.7	20.32	20.14	20.6	0.068	0.56
		25	24.3	24.6	25	25.3	−0.13	0.39

Test 3	Conductivity (Us/Cm)	300	303.4	297.6	301.9	302.6	0.042%	0.12%
		450	457.9	452.8	450.9	452.9	0.13%	0.22%
		500	508.4	505.9	495.7	504.9	0.15%	0.28%

Test 4	Dissolved oxygen (Mg/L)	3.0	3.04	3.08	3.02	2.91	0.08%	0.36%
		5.0	5.07	5.01	5.15	5.05	0.43%	0.54%
		6.0	6.15	6.02	6.17	6.09	0.55%	0.65%

## Data Availability

The data used to support the findings of this study are included within the article.
